# CDK4 and miR-15a comprise an abnormal automodulatory feedback loop stimulating the pathogenesis and inducing chemotherapy resistance in nasopharyngeal carcinoma

**DOI:** 10.1186/s12885-016-2277-2

**Published:** 2016-03-18

**Authors:** Zhen Liu, Chao Cheng, Xiaojun Luo, Qiong Xia, Yejie Zhang, Xiaobing Long, Qingping Jiang, Weiyi Fang

**Affiliations:** Third Affiliated Hospital of Guangzhou Medical University, Guangzhou, 510150 PR. China; Cancer Research Institute, Southern Medical University, Guangzhou, 510515 China; Cancer Center, Traditional Chinese Medicine-Integrated Hospital, Southern Medical University, Guangzhou, Guangdong 510315 China; Department of Pathology, Basic School of Guangzhou Medical University, Guangzhou, 510182 China; Pediatric Center of Zhujiang Hospital, Southern Medical University, Guangzhou, 510282 PR. China; Otorhinolaryngology of Zhujiang Hospital, Southern Medical University, Guangzhou, 510282 PR. China

**Keywords:** NPC, CDK4, miR-15a, Tumor suppressor

## Abstract

**Background:**

In previous investigation, we reported that stably knocking down cyclin-dependent kinase 4(CDK4) induced expression of let-7c, which further suppressed cell cycle transition and cell growth by modulating cell cycle signaling in nasopharyngeal carcinoma (NPC). In this study, we further explored the molecular function and mechanism of CDK4 modulating miRNAs to stimulate cell cycle transition, cell growth, and Cisplatin (DDP) -resistance on in NPC.

**Methods:**

We identified changes in miRNAs by miRNA array and real-time PCR and the effect on DDP after knocking down CDK4 in NPC cells. Further, we investigated the molecular mechanisms by which CDK4 modulated miR-15a in NPC. Moreover, we also explored the role of miR-15a and the effect on DDP in NPC. Finally, we analyzed the correlation of miR-15a and CDK4 expression in NPC tissues.

**Results:**

In addition to let-7 family members, we observed that upregulated expression of miR-15a was significantly induced in CDK4-suppressed NPC cells. Further, we found that knocking down CDK4 suppressed c-Myc expression, and the latter directly suppressed the expression of miR-15a in NPC. Furthermore, miR-15a as a tumor suppressor antagonized CDK4 repressing cell cycle progression and cell growth in vitro and in vivo and induced the sensitivity of cells to DDP by regulating the c-Myc/CCND1/CDK4/E2F1 pathway in NPC. Finally, miR-15a was negatively weak correlated with the expression of CDK4 in NPC.

**Conclusions:**

Our studies demonstrate that CDK4 and miR-15a comprise an abnormal automodulatory feedback loop stimulating the pathogenesis and inducing chemotherapy resistance in NPC.

**Electronic supplementary material:**

The online version of this article (doi:10.1186/s12885-016-2277-2) contains supplementary material, which is available to authorized users.

## Background

Cell cycle progression is controlled in part by a family of cyclin proteins and cyclin dependent kinases (Cdks). CDK4 is a member of cyclin-dependent kinase family, and in complex with D-type cyclins, is thought to regulate cell growth during cell cycle transition from G1 to S phase. In previous studies, CDK4 was reported to play a significant role in promoting the pathogenesis of tumors including oral squamous cell carcinoma [1], pancreatic endocrine tumors [2], lung cancer [3, 4], nasopharyngeal carcinoma [5–7], and other tumors [8–10].

MicroRNAs (miRNAs) are ~22-nucleotide (nt) small RNAs that have emerged as important factors regulating deadenylation, translation, and decay of their target mRNAs. In recent years, many miRNAs were observed to be deregulated and participate in the carcinogenesis by modulating important tumor-associated genes [11–15]. miR-93, derived from miR-106b-25 cluster, is elevated in various types of cancers and plays oncogenic roles by suppressing significant tumor suppressors including PTEN, LATS2, and TGFBR2 et al. [16]. miR-18b is a potential oncogene suppressed by CTGF through PI3K/AKT/c-Jun/c-Myc to induce cell growth [17]. miR-184 induced by PDCD4 directly suppressed c-Myc and Bcl-2, which inhibited cell growth and stimulated cell apoptosis in nasopharyngeal carcinoma [18].

NPC is one of the most common carcinomas with a malignant phenotype in Southern China and Southeast Asian countries. Synergetic contributions of viral infections, genetic alterations, and environmental factors drive the aberrant activity of a variety of genes, which stimulate the initiation and development of NPC. In previous investigation, we have reported that overexpressed CDK4 was considered an unfavorable factor associated with NPC progression and poor prognosis. Knocking down CDK4 induced the upregulation of let-7c and the latter further reduced cell cycle progression and cell growth by modulating p16/CDK4/E2F1 signaling in NPC. This demonstrated the significance of miRNA regulation of CDK4 in NPC pathogenesis [6]. In this study, we further study the molecular basis of CDK4 modulating miRNAs in inducing cell cycle transition, cell proliferation, and the effect on DDP in NPC.

## Methods

### Sample collection and cell culture

Two NPC cell lines 5–8 F and HONE1 as well as shCDK4-2 and shCDK4-3 [6] were obtained from Cancer Research Institute of Southern Medical University and maintained in RPMI 1640 medium supplemented with 10 % newborn calf serum (NBCS) (PAA Laboratories, Inc, Pasching, Austria) in a humidified chamber with 5 % CO_2_ at 37 °C. All 63 fresh NPC and 15 NP samples (13 cases for chronic nasopharyngitis tissuses and 2 cases for normal nasopharyngeal tissues) were obtained from an otorhinolaryngologist using nasal endoscope. Subsequently, all samples were immediately stored in liquid nitrogen. Clinical processes were approved by the Ethics Committees of People’s Hospital of Zhongshan City and patients gave informed written consent.

### miRNA array for shCDK4

In-house two-channel oligo-arrays (CCDTM-miRNA850-V4px) from NIH including 713 human, mammalian, and viral mature antisense miRs plus two internal controls with seven serial dilutions were endowed by Professor Wang E and Marincola FM. Six to seven microgram total RNA samples isolated respectively from shCDK4 and its control 5-8F cells were labeled by Cy5-dCTP and Cy3-dCTP, respectively, in a reverse transcription reaction. The balanced mixture of Cy5- and Cy3-labeled targets was co-hybridized against miRNAs chip. The experiments were repeated four times and scanned images were converted to digital data by GenePixpro V6.0 (Molecular Devices Corporation, Sunnyvale, CA, USA). Finally, the data were analyzed using BRB ArrayToolsV3.7.2 software (National Cancer Institute, Bethesda, MD, USA).

### RNA isolation and qRT-PCR

RNA was extracted from NPC cell lines, NPC tissues and normal nasopharynx tissues using Trizol (Takara, Shiga, Japan). For miR-15a qRT-PCR expression analysis, mature miRNAs were reverse-transcribed, and real-time PCR was performed using All-in-One™ miRNA qRT-PCR Detection Kit following the manufacturer’s protocol. (GeneCopoeia™, Cat.No: AOMD-Q020). All data were normalized to U6 expression. For CDK4 qRT-PCR, RNA was transcribed into cDNA and amplified with specific sense/antisense primer [7]. The assays were performed in accordance with manufacturer’s instructions (Takara, Shiga, Japan). The PCR reaction for each gene was repeated three times. miRNA and mRNA expression was normalized to U6 and ARF5, respectively using the 2-ΔΔCt method as previously described [6]. Expression values (2^-ΔΔCt^) of CDK4 or miR-15a in NPC tissues greater than or equal to the mean expression value of NP tissues were considered high expression. Conversely, expression values of CDK4 or miR-15a in NPC tissues less than NP tissues were regarded as low expression.

### Western blot analysis

Western blot was carried out according to previous descriptions [17, 18] with rabbit polyclonal CDK4, GAPDH, E2F1 antibody (1:400; Santa Cruz Biotechnology, Santa Cruz, USA); C-Myc antibody (Cell signaling technology, Danvers, USA), and CCND1 antibody (1:500; Epitomics, Burlingame, USA). An HRP-conjugated anti-rabbit IgG antibody was used as the secondary antibody (Zhongshan, Beijing, China). Signals were detected using enhanced chemiluminescence reagents (Pierce, Rockford, IL) and Bio-RAD ChemiDox XRS.

### Chromatin immunoprecipitation assay

Chromatin immunoprecipitation assay was carried out according to previous descriptions [12, 13]. DNA–protein complexes were immunoprecipitated from 5-8F and HONE1 cells with the transfection of c-Myc cDNA by using the Chromatin Immunoprecipitation Kit (Millipore, Billerica, MA, USA), according to the manufacturer’s protocol with 1 mg polyclonal c-Myc antibody or 1 mg normal mouse IgG (Millipore). Precipitated DNA was subjected to PCR analysis using specific primers (Forward:5′AAATGCCTGTGGGCTGGTAGCT3′; Reverse: 5′GCCGCGGAGGTGAAGTGAACT3′) to amplify across the DLEU2/miR-15a promoter region [19]. Finally, DNA was analyzed by 1 % agarose gel electrophoresis.

### Luciferase activity assay

The plasmids including pGL3-control and pGL3-promoter used for luciferase reporter gene expression analysis were bought from Promega Ltd. pGL3-Wild DLEU2 1A promote vector(pGL3-W) containing c-Myc binding site (CACGTG) was constructed by RT-PCR using specific primers(Forward:5′AA*GAGCTC(Sac I)*AAGCCGGCAGGGCGGTTTT3′;Reverse: 5′AA*CTCGAG(XhoI)*TACCGAC TGCGCCAGCCTTG3′). Meanwhile, pGL3-Mutant vector with a mutated c-Myc binding site (CGCATT) in the DLEU2 regulatory region was also constructed. 5-8F cells with exogenous c-Myc expression were plated in 24-well plates at a density of 1 × 10^4^ cells/well. After 24 h, pGL3-C pGL3-W or pGL3-M were respectively transfected with pcDNA3.1/c-Myc or its control vector were introduced into 5-8F cells using Lipofectamine 2000. After 48 h, firefly luciferase activity was measured using the dual luciferase reporter assay system according to the manufacturer’s protocol.

### Transient transfection with miR-15a mimics and its inhibitor

miR-15a mimic and its inhibitor were designed and synthesized by Guangzhou RiboBio (RiboBio Inc, China). Twenty-four hours prior to transfection, NPC cells were plated onto a 6-well plate or a 96-well plate (Nest, Biotech, China) at 30–50 % confluence. They were then transfected into cells using TurboFectTM siRNA Transfection Reagent (Fermentas, Vilnius, Lithuania) according to the manufacturer’s protocol. Cells were collected after 48–72 h for further experiments.

### miRNA target validation

CCND1 were predicted to be directly regulated targets of miR-15a miRwalk softwares (University of Heidelberg, Mannheim, Germany). A 289 fragment of CCND1 3′UTR amplified by PCR primers (Sense:5′-AA*CTCGAG*CCATTTTCTTATTGCGCTGC-3′; Antisense:5′-AA*GCGGCCGC*GGCTAAGTGAAGCATGAGGT-3′) was cloned into psiCHECK-2 vectors (named wt) with XhoI and NotI restriction enzyme sites. Site-directed mutagenesis of the miR-15a binding site in CCND1 3′UTR was performed using GeneTailor Site-Directed Mutagenesis System (Invitrogen; named mt). For reporter assays, wt or mt vector and the control vector psiCHECK-2 vector were cotransfected into SUNE1 cells with miR-15a mimics or inhibitor. Luciferase activity was measured at 48 h after transfection using the Dual-Luciferase Reporter Assay System (Promega Corporation, Madison, WI, USA).

### Cell proliferation analysis

Cell proliferation was analyzed using MTT assay as described previously [17, 18]. For miR-15a inhibitor and mimics, the cells were incubated for 1, 2, or 3 days.

### Cell cycle assay

To evaluate cell cycle distribution, cells were fixed in 70 % ice-cold ethanol for 48 h at 4 °C, and stained by incubating cells with PBS containing 10 μg/mL propidium iodide and 0.5 mg/mL RNase A for 15 min at 37 °C, and analyzed for the DNA content of labeled cells by FACS Caliber Cytometry (BD Bioscience, USA). Each experiment was done in triplicate.

### Establishment of NPC cell line with stable expression of miR-15a

Lentivirus (GV209) particles carrying hsa-pri-miR-15a precursor and its control were prepared. Lentiviral transduction of 5–8 F and HONE1 cells was carried out according to the manufactures’ protocol(Genechem Company, Shanghai, China). The resulting cells were seeded onto 96-well plates and cultured for 3 weeks to produce a stable miR-15a-overexpressing 5-8F and HONE1 cells and their respectively control cells. High expression of miR-15a was validated by qRT-PCR.

### In vivo tumorigenesis in nude mice

A total of 1 × 10^6^ logarithmically growing miR-15a-overexpressing 5-8F and HONE1 cells and their control cells in 0.1 ml RPMI 1640 medium were respectively subcutaneously injected into the left or right flank of 4–6-week-old male BALB/c nu/nu mice (*N* = 5). Mice were maintained in a barrier facility on HEPA-filtered racks and fed with an autoclaved laboratory rodent diet. All animal studies were conducted in accordance with the principles and procedures outlined in Southern Medical University Guide for the Care and Use of Animals. After 25 days the mice were killed, and tumor tissues were excised and weighted.

### MTT cytotoxicity assay

NPC Cells (5-8F and HONE1) with miR-15a overexpression or their control cells were respectively seeded in 96-well plates in 100 μl DMEM medium supplemented with 10 % FBS at 5 × 10^3^ cells/well. Once the cells attached, they were respectively treated with DDP in 2.5, 5, 10, 20, 30, 40 or 50 μM (0.5 mg/ml) and incubated at 37 °C in 5 % CO_2_ for 48 h. Subsequently, 10 μl of MTT (5 mg/ml) (Sigma, StLouis, MO, USA) was added to each well, and the plates were incubated at 37 °C for 4 h. Further, the supernatants were removed and 100 μl of DMSO (Sigma) was added to each well. The absorbance value (OD) of each well was measured at 490 nm and half maximal inhibitory concentration (IC50) was calculated. Experiments were performed three times.

### Statistical analysis

All data were analyzed for statistical significance using SPSS 19.0 software. The Student’s test was applied to examine the differences of mRNA expressions of CDK4 and miR-15a between normal epithelium and cancer tissues of nasopharynx. The relationship between CDK4 and miR-15a expression levels was analyzed using pearson test. Two-tailed Student’s *t*-test was used for comparisons of two independent groups. One-way ANOVA was used to determine the differences between groups for all in vitro analyses. A *P* value of less than 0.05 was considered statistically significant.

## Results

### Stably downregulated CDK4 expression induced the expression of miR-15a in vitro in NPC

In a previous study, we demonstrated that suppressing CDK4 expression using lentiviral-mediated shRNA inhibited NPC cell proliferation and G1 to S cell cycle transition by inducing let-7c. To further investigate the effect of CDK4 on miRNAs in NPC, we used miRNA chip to compare the differential miRNA expression between shCDK4-2 and shCDK4-3 and mock cells [6]. We observed that knocking down CDK4 significantly stimulated the expression of miR-15a and let-7 family members including let-7c (Fig. 1a). Further, we validated the upregulated expression of miR-15a in CDK4-suppressed 5-8F NPC cells by real-time qPCR (Fig. 1b).

**Fig. 1:** Stable suppression of CDK4 elevated the expression of miR-15a in NPC. **a**. The expression of miR-15a and let-7 family members was induced after stable knockdown of CDK4 NPC cells based on a micro-RNA array assay. **b**. miR-15a expression was significantly increased in NPC cells with stably knocking down CDK4 expression by qPCR assay. (*P < 0.05)

### Transiently knocking down CDK4 also elevated the expression of miR-15a

To confirm that CDK4 knockdown elevated miR-15a expression in NPC, we used siRNA-CDK4 to transfect NPC 5-8F and HONE1 cells. We observed that siCDK4-2 provided the greatest suppression of CDK4 mRNA (Fig. 2a) among three siCDK4 fragments tested in NPC 5-8F and HONE1 cells. Further, we validated that siCDK4-2 significantly downregulated CDK4 protein levels in NPC 5-8F and HONE1 cells (Fig. 2b). Finally, we found that transiently knocking down CDK4 by siRNA also stimulated the expression of miR-15a (Fig. 2c).

**Fig. 2:** Transiently inhibited CDK4 by siRNA stimulated the expression of miR-15a. **a**. The interference efficiency of siCDK4s in mRNA level was examined by qPCR in NPC cells. **b**. Western blot was used to validate the interference efficiency of siCDK4-2 on protein levels in NPC cells. **c**. Transiently inhibited CDK4 stimulated the expression of miR-15a by qPCR. (*P < 0.05)

### Inhibition of CDK4 induced miR-15a expression by suppressing c-Myc expression

In a previous report, we found that inhibition of CDK4 decreased the expression of CCND1,CDK6, and E2F1 [6]. Here, we observed that stably knocking down CDK4 reduced the expression of c-Myc in NPC 5-8F cells (Fig. 3a). Further, we observed that suppressing expression of c-Myc (Fig. 3b) markedly increased the expression of miR-15a in NPC 5-8F and HONE1 cells (Fig. 3c).

**Fig. 3:** Knocking down CDK4 induced miR-15a expression by suppressing c-Myc expression. **a**. Stable suppression of CDK4 reduced the expression of c-Myc in NPC cells. **b**. si-Myc inhibited the expression of c-Myc in NPC cells. **c**. Transiently inhibited c-Myc by siRNA stimulated the expression of miR-15a. (*P < 0.05)

### c-Myc directly binds to the promoter of miR-15a (DLEU2)

Atrributing to the fact that the miR-15a promoter contains a binding site for c-Myc, we speculated that c-Myc negatively modulate miR-15a expression. To test this, c-Myc was transfected into NPC 5-8F and HONE1 cells. The results indicated that c-Myc was highly expressed in NPC cells compared to mock cells (Fig. 4a). Further, overexpressed c-Myc significantly reduced the expression of miR-15a in NPC 5-8F and HONE1 cells. Finally, chromatin immunoprecipitation combined with PCR analysis (Fig. 4c) and luciferase reporter assay (Fig. 4d) were used to confirm that c-Myc could directly bind its promoter in NPC.

**Fig. 4:** c-Myc binds to the promoter of miR-15a in NPC cells. **a**. c-Myc cDNA was transfected to 5–8 F and HONE1 NPC cells and its protein expression was examined by western blot. **b**. Overexpressed c-Myc reduced the expression of miR-15a in NPC cells. **c**. Crosslinked chromatin preparation from mock and pcDNA3.1-C-Myc transfected 5-8F and HONE1 cells was immunoprecipitated with anti-C-Myc. The c-Myc binding sites on the immunoprecipitated DNA was determined by PCR. Amplification of input chromatin (input) before immunoprecipitation was served as positive controls for chromatin extraction and PCR amplification. Chromatin immunoprecipitation using normal human IgG served as a negative control. The result indicated that overexpressed c-Myc could bind more miR-15a promoter region than that in control group in NPC cells. **d**. Luciferase reporter assay indicated that c-Myc could directly bind miR-15a promoter in NPC. (*P < 0.05)

### miR-15a suppresses cell proliferation and cell cycle progression in vitro and in vivo in NPC

To investigate the effect of miR-15a on NPC, we introduced miR-15a mimics into NPC 5–8 F and HONE1 cells. Compared to negative controls, we found that miR-15a mimics inhibited cell growth and cell cycle progression from G1 to S and G2 in vitro in NPC cells by MTT (Fig. 5a, b) and cytometry assays (Fig. 5c, d). Further, we established stable overexpression of miR-15a in NPC 5-8F and HONE1 cells using lentiviral infection (Additional file 1: Figure S1). An in vivo tumorigenesis study inoculating these cells into nude mice showed that the average tumor weight was significantly decreased in miR-15a-overexpressing xenografts compared with their respectively controls (Fig. 5e).

**Fig. 5:** miR-15a suppressed cell cycle progression and cell growth in NPC. **a** and **b**. miR-15a mimics inhibited cell proliferation in NPC 5-8F and HONE1 cells by MTT assay. **c** and **d**. miR-15a mimics blocked cell cycle progression from G1 to S phase in NPC 5-8F and HONE1 cells. **e**. Lentivirus-mediated expression of miR-15a suppressed tumorigenesis of NPC 5-8F and HONE1 cells in vivo in nude mice. **f** and **g**. miR-15a inhibitor partially restored cell proliferation in CDK4-suppressed NPC cells. (*P < 0.05)

### miR-15a antagonizes the action of CDK4 in NPC

To investigate the effect of miR-15a on CDK4 in NPC, we introduced miR-15a inhibitor into CDK4-suppressed NPC cells (shCDK4-2 and 3). We observed that suppression of miR-15a using inhibitor (Additional file 2: Figure S2) partially restored the cell proliferative ability (Fig. 5f, g). Our results demonstrated that miR-15a is a potential tumor suppressor in NPC.

### miR-15a suppresses c-Myc/CCND1/CDK4/E2F1 pathway in NPC

In a previous investigation, miR-15a was reported to directly target CCND1, thereby suppressing tumor cell growth [20, 21]. In this study, we found that miR-15a mimics not only reduced CCND1 expression, but also suppressed the expression of c-Myc, CDK4 and E2F1 in NPC 5-8F and HONE1 cells (Fig. 6a). Our results suggest a feedback loop between CDK4 and miR-15a.

**Fig. 6:** miR-15a modulated cell cycle signaling in NPC. **a**. miR-15a mimics decreased the expression of key cell cycle transition factors including c-Myc, CCND1,CDK4, and E2F1. **b**. Luciferase reporter assay was used to determine miR-15a directly targeting the 3′UTR of CCND1. (*P < 0.05)

### miR-15a directly targeting CCND1

To further study the mechanism of miR-15a suppressing cell proliferation, we explored its directly target gene in NPC. Interestingly, CCND1 was predicted as the directly target gene by bioinformatics assay. We observed that Wild-type (wt) or mutant (mt) 3′UTR vector of CCND1 and miR-15a mimics or inhibitor NPC cells were cotransfected with NPC SUNE1 cells. The results showed a significant decrease of luciferase activity in wt vector transfected with miR-15a mimics (Fig. 6b, lanes 1; *P* < 0.001) or an obvious increase of luciferase activity by using miR-15a inhibitor (Fig. 6b, lanes 3; *P* < 0.001) when compared with miR control, whereas the activity of mt vector was unaffected (Fig. 6b, lanes 5 and 6) by using miR-15a mimics or inhibitor. Taken together, these results strongly supported that CCND1 was the direct targets of miR-15a in NPC cells.

### Silencing of CDK4 and ovexpressed miR-15a respectively enhance DDP chemosensitivity to NPC cells in vitro and in vivo

The NPC cell line stably downregulating CDK4 exhibited significantly increased sensitivity to DDP. The results indicated that the IC50 of DDP was 28.43 μM in the parental NPC 5–8 F cells, whereas reduced to 16.12 μM in CDK4 silencing NPC 5–8 F cells (Fig. 7a). Further, we evaluated the effectiveness of DDP in miR-15a-overexpressed NPC 5–8 F cells. The results showed that IC50 value was significantly reduced in miR-15a-overexpressed NPC cells (14.40 μM) compared with the control cells treated with DDP (31.43 μM).

**Fig. 7:** Knocking down CDK4 or increased miR-15a induced the sensitivity of NPC cells to DDP. **a**. Knocking down CDK4 elevated the sensitivity of NPC cells to DDP. **b**. Overexpressed miR-15a stimulated the increased sensitivity of NPC cells to DDP

### CDK4 mRNA expression is negatively weak correlated with expression of miR-15a

Due to the existence of feedback regulation loop between CDK4 and miR-15a, we speculated that CDK4 expression is negatively correlated with expression of miR-15a. To confirm this hypothesis, we examined the expression of CDK4 mRNA and miR-15a in NPC and NP tissues. There was an increased tendency of CDK4 mRNA in NPC tissues compared to NP tissues (*P* = 0.0920) (Fig. 8a). On the contrary, miR-15a was downregulated expression in NPC tissues compared to NP tissues (*p* = 0.0323) (Fig. 8b). Further, a significantly inverse weak correlation was observed between CDK4 mRNA and miR-15a expression in NPC tissues (Fig. 8c).

**Fig. 8:** The increased expression of CDK4 mRNA was negatively weak correlated with the reduced miR-15a expression in NPC. **a**. CDK4 mRNA was upregulated in NPC tissues compare to NP tissues. **b**. miR-15a expression was upregulated in NPC tissue compare to NP tissues. **c**. CDK4 mRNA was negatively weak correlated with the expression of miR-15a in NPC

## Discussion

CDK4 is a member of the cyclin-dependent kinase family and a key factor for cell cycle signaling during transition from G1 to S phase. CDK4overexpression has been observed in many tumor types, including NPC. In previous report, we had observed that knocking down CDK4 induced let-7c through cell cycle signaling, and let-7c in turn suppressed cell proliferation and cell cycle progression by modulating p15/p16/CDK4/E2F1 [6]. This study suggested that CDK4 promoted NPC pathogenesis by modulating miRNAs. However, CDK4-mediated miRNAomics linking to the initiation and development of NPC had not been investigated.

In this study, we used miRNA array to observe the differential expression of miRNA in CDK4-suppressed NPC cells. Interestingly, let-7 family members including let-7c reported by us [6] were shown to be elevated expression after knocking down CDK4 NPC cells. Tumor suppressor miR-15a was also observed to be upregulated in CDK4-suppressed NPC cells. Further, we confirmed the increased expression of miR-15a after stably or transiently knocking down CDK4 NPC cells by qPCR, which demonstrated that CDK4 negatively modulates the miR-15a expression in NPC.

In previous study, we demonstrated that CDK4 induced the expression of transcription factor E2F1 by modulating CCND1, CDK6, p21, and pRB in NPC cells [6]. Because E2F1 directly binds to the promoter of c-Myc and stimulates the expression of c-Myc [22], we speculated that CDK4 positively regulates c-Myc expression in NPC. Consistent with this expectation, we observed downregulated expression of c-Myc after knockdown of CDK4 in NPC cells.

c-Myc is an key oncogenic transcription factor promoting cellular proliferation and cancer stemness in NPC [23, 24]. Furthermore, our recent studies indicated that c-Myc directly modulated the expression of miR-184 and miR-18b participating in the pathogenesis of NPC [17, 18]. In previous study, c-Myc had been reported to directly bind to the promoter of DLEU2 gene which encompasses the tumor suppressor miR-15a. This binding in turn decreases expression of both DLEU2 and miR-15a [25]. We speculated that upregulation of miR-15a mediated by CDK4 suppression was at least in part modulated by c-Myc in NPC. We used siRNA to knock down c-Myc and observed that the expression of miR-15a was significantly increased in NPC cells. Further, we utilized chromatin immunoprecipitation combined with qPCR assays and found that c-Myc directly bind to the miR-15a promoter in NPC. Furthermore, we observed the significant reduction of luciferase activity in c-Myc-binded miR-15a promoter. Our investigation demonstrated that c-Myc directly suppressed the expression of miR-15a in NPC cells.

miR-15a has been identified as a tumor suppressor in some tumor types [20, 21, 26–32]. However, its role in NPC has not been yet reported. In this study, we found that miR-15a inhibited cell cycle progression from G1 to S phase and cell growth in vitro and in vivo in NPC cells. We also observed that miR-15a inhibitor partially restored cell growth in CDK4-suppressed NPC cells. These results demonstrated that miR-15 functions as a tumor suppressor and could overcome the action of CDK4 in NPC.

In previous reports, miR-15a had been reported to directly suppress the expression of Sox5, which induced the blockage of cell growth, migration, and invasion in pituitary tumors. Furthermore, miR-15a directly targets Cripto, Bmi-1, CCNE1, RECK, VEGF, CCND1, and BCL-2 to suppress the malignant phenotypes in various tumors including NSCLC, pancreatic ductal adenocarcinoma, breast cancer, neuroblastoma, multiple myeloma, and osteosarcoma [20–22, 25–32]. However, the molecular basis of miR-15a has never been reported in NPC. In this study, miR-15a was observed to block cell cycle transition at G1/S, which was a key factor inducing cell growth arrest in NPC. We suspected that miR-15a mediated the suppression of NPC cell growth based on its modulation of cell cycle factors. We observed that miR-15a not only directly inhibited the expression of CCND1, one its known direct targets, but also downregulated the expression of CDK4, c-Myc, and E2F1. These results demonstrated that miR-15a suppressed cell growth through c-Myc/CCND1/CDK4/E2F1 signaling in NPC. More interestingly, a positive feedback loop of CDK4-c-Myc-miR-15a was observed, which was similar to our previous report for CTGF-C-Jun/C-Myc-miR-18b and CDK4-E2F1-let-7c which promotes NPC pathogenesis [6, 17].

Cell cycle arrest is a key factor that usually induced the elevation of chemotherapy sensitivity in tumor [33–35]. In this study, we observed that knocking down CDK4 and overexpressed miR-15a significantly induced the chemotherapy sensitivity of DDP by inhibiting cell cycle progression, which hinted the negatively abnormal feedback loop between CDK4 and miR-15a as an important signal resisting chemotherapy in NPC pathogenesis.

We have previously reported increased expression of CDK4 in NPC [5–7]. However, the correlation between CDK4 expression and miR-15a has not been documented. In this study, we observed elevated CDK4 mRNA and decreased expression of miR-15a in NPC tissues compared to nasopharynx tissues. Further, we found that CDK4 mRNA expression was negatively weak correlated with the expression of miR-15a in NPC tissues.

## Conclusions

In summary, our study demonstrated that knocking down CDK4 induced the activation of miR-15a by modulating the CDK4/E2F1/c-Myc pathway. This in turn suppressed cell proliferation and inducing chemotherapy sensitivity by controlling c-Myc/CCND1/CDK4/E2F1 signaling, and suggested an abnormal automodulatory feedback loop of CDK4-c-Myc-miR-15a which promoted NPC pathogenesis and acquired DDP resistance.

## Additional files

Additional file 1: Figure S1. Lentivirus-mediated miR-15a expression in NPC 5–8 F and HONE1 cells. (TIFF 342 kb) Additional file 2: Figure S2. Specific inhibitor of miR-15a was used to inhibit the expression of miR-15a in shCDK4-2 and shCDK4-3 NPC 5–8 F cells. (TIFF 383 kb)

## Abbreviations

NPC: nasopharyngeal carcinoma
DDP: cisplatin
CDK4: cyclin-dependent kinase 4
miRNAs: microRNAs
qRT-PCR: quantitative reverse transcription-PCR
IC50: half maximal inhibitory concentration
DNA: deoxyribonucleic acid
MTT: 3-(4,5)-dimethylthiahiazo (−z-y1)-3,5-di- phenytetrazoliumromide
DMSO: dimethyl sulfoxide
ANOVA: analysis of variance
